# M2 macrophage polarization in systemic sclerosis fibrosis: pathogenic mechanisms and therapeutic effects

**DOI:** 10.1016/j.heliyon.2023.e16206

**Published:** 2023-05-12

**Authors:** Mingyue Hu, Zhongliu Yao, Li Xu, Muzi Peng, Guiming Deng, Liang Liu, Xueyu Jiang, Xiong Cai

**Affiliations:** a Department of Rheumatology of the First Hospital and Institute of Innovation and Applied Research in Chinese Medicine, Hunan University of Chinese Medicine, Changsha, Hunan 410208, China; b State Key Laboratory of Dampness Syndrome of Chinese Medicine, The Second Affiliated Hospital of Guangzhou University of Chinese Medicine, Guangzhou, 510000, China; c Yueyang Hospital of Chinese Medicine, Hunan University of Chinese Medicine, Yueyang, Hunan 414000, China

**Keywords:** Systemic sclerosis, Fibrosis, M2 macrophage polarization, Fibroblasts, Myofibroblasts

## Abstract

Systemic sclerosis (SSc, scleroderma), is an autoimmune rheumatic disease characterized by fibrosis of the skin and internal organs, and vasculopathy. Preventing fibrosis by targeting aberrant immune cells that drive extracellular matrix (ECM) over-deposition is a promising therapeutic strategy for SSc. Previous research suggests that M2 macrophages play an essential part in the fibrotic process of SSc. Targeted modulation of molecules that influence M2 macrophage polarization, or M2 macrophages, may hinder the progression of fibrosis. Here, in an effort to offer fresh perspectives on the management of scleroderma and fibrotic diseases, we review the molecular mechanisms underlying the regulation of M2 macrophage polarization in SSc-related organ fibrosis, potential inhibitors targeting M2 macrophages, and the mechanisms by which M2 macrophages participate in fibrosis.

## 1 Introduction

Systemic sclerosis (SSc), also termed scleroderma is an orphan disease characterized by autoimmunity, fibrosis of the skin and internal organs, and vasculopathy [1,2]. Various cell types are thought to be involved in the pathogenesis of SSc, Numerous investigations into inflammatory cells and their mediators have revealed that macrophages are crucial to the occurrence and progression of SSc fibrosis [[3], [4], [5]]. Skin biopsies have revealed increased infiltration of inflammatory cells, primarily CD14^+^ monocytes/macrophages, in newly occurring SSc skin fibrosis [6]. In an independent cohort study, the gene expression signature associated with blood-derived human SSc macrophages was found to be enriched in SSc skin and was correlated with skin fibrosis [7]. Fibroblasts are key effector cells of the fibrotic response, and in limited cutaneous systemic sclerosis (lcSSc), the percentage of circulating fibroblasts is positively correlated with skin thickness [8], and the heterogeneity of gene expression in fibroblasts determines the functional Heterogeneity, which evolves with disease progression [9,10]. *In vitro* studies have shown that the coculture of SSc macrophages with fibroblasts resulted in fibroblast activation [7]. Additionally, soluble CD163 (sCD163), a marker of M2 macrophages [11], is abundant in the circulation of patients with SSc [12], and the infiltration of CD163^+^ macrophages is upregulated in fibrotic skin and lungs [13,14]. This reveals an inextricable link between M2 macrophages and SSc fibrosis, and further study and discussion of M2 macrophages in SSc may provide new insights into the pathogenesis and therapeutic studies of SSc.

## 2 SSc and M2 macrophages

### 2.1 Overview of SSc

SSc is a complex immune-mediated multi-organ connective tissue disease of unknown etiology. It is an extraordinary circumstance that primarily affects young and middle-aged women, severely damaging their quality of life and leading to disproportionate morbidity and mortality [15,16]. Furthermore, SSc contains a broad group of conditions with wildly differing clinical symptoms, natural histories, treatment responses, and outcomes. There are currently no authorized disease-modifying therapies for SSc [17]. The pathogenesis of SSc is not completely understood but contains a triad of hallmarks, including immune dysfunction, vasculopathy, and fibrosis [18]. Injury to endothelial cells (EC) is suggested as a key initiating event that causes vascular remodeling with capillary damage, intimal arteriole proliferation, and ultimately blood vessel occlusion [19]. The current model for SSc pathogenesis proposes that unknown etiologic factors initiated a chain of pathogenetic events in a genetically susceptible host, triggering microvascular injury marked by structural and functional endothelial cell abnormalities [20] (Fig. 1). It is widely assumed that SSc is driven by a complicated interaction of genetic and environmental factors. In individuals liable to epigenetic and genetic factors, certain environmental factors may impair ECs, resulting in vascular remodeling, aberrant inflammation, and the progression of SSc [21]. In addition to environmental factors, autoimmune attacks of γδT cells and anti-endothelial cell antibodies (AECAs) contribute to the immune system-driven initial vascular injury [22]. EC dysfunction increases the production and release of a plethora of potent immune mediators, including chemokines, cytokines, polypeptide growth factors, and a variety of other substances [20]. In response to these mediators, immune cells are recruited from the bloodstream and bone marrow, generate a perivascular infiltrate, and secrete cytokines and growth factors, leading to prolonged inflammation [20]. The main cell type responsible for the excessive production of collagen and other extracellular matrix components, myofibroblasts, are activated by chronic inflammation, which results in tissue fibrosis [23].

**Fig. 1:** Overview of the pathogenesis of SSc. A complex interaction between the vasculature, immune cells, and fibroblasts triggers and reinforces the onset and progression of SSc, which in turn causes vasculopathy, inflammation, autoimmunity, and an excessive buildup of ECM. Genetic and environmental factors are responsible for aberrant ECs. Chemokines and cytokines generated by the aberrant ECs recruit leukocytes. Local fibroblasts, ECs, and fibrocytes are activated and differentiated as a result of the pro-fibrotic growth factors and cytokines secreted by activated T cells, B cells, and macrophages. DAMPs, damage-associated molecular patterns; ROS, reactive oxygen species.

### 2 2 Macrophage polarization

It is noteworthy that macrophages can sense their microenvironment and change how they behave through phenotypic plasticity. Macrophages perform their duties by changing their phenotype in response to stimuli from the tissue around them. This plasticity, which is also referred to as M1/M2 macrophage polarization, is the outcome of a carefully orchestrated process that leads to the differential expression of surface markers, the production of particular factors, and the execution of biological activities.

Macrophages are important cells that perform innate and adaptive immune functions and are found in almost all tissues. Classically activated macrophages (M1) and alternatively activated macrophages (M2) are the two main types of macrophages [24,25]. M1 macrophages are induced by interferon-γ (IFN-γ) and lipopolysaccharide (LPS). M1 macrophages express co-stimulatory molecules CD80, CD86, and *MHC* class *II* molecules (*MHC-II*), and secrete high levels of pro-inflammatory cytokines and mediators, including interleukin-1β (IL-1β), IL-6, tumor necrosis factor-α (TNF-α), and inducible nitric oxide synthase (iNOS), etc. [26]. M1 macrophages are antigen-presenting cells, promoting inflammation and Th1 immune response in response to foreign pathogens and tumor cells while mediating reactive oxygen species (ROS)-induced tissue damage and impairing wound healing and tissue regeneration [26,27]. IL-4, IL-13, IL-10, transforming growth factor-β (TGF-β) immune complexes, complements, and apoptotic cells can all trigger M2 polarization [24]. M2 macrophages are highly phagocytic, and they produce TGF-β, IL-10, vascular endothelial growth factor (VEGF), and other regulatory factors and reduce inflammation, improve wound healing, regulate the immune response and angiogenesis, and stimulate extracellular matrix (ECM) generation [28] (Fig. 2). M2 macrophages are classified as M2a [29,30], M2b [[31], [32], [33]], M2c [32,34], and M2d [35,36] (Fig. 2).

**Fig. 2:** Inducible factors, phenotypes, and functions of the different subtypes of macrophages. Natural macrophage (M0) differentiates to M1 and M2, which is driven by different inducible factors. The M2 macrophages are further classified as M2a, M2b, M2c, and M2d, relative to their secreted cytokine profiles and complex functions. CXCL-1, The chemokine (C-X-C motif) ligand-1; CCL-1, C–C motif chemokine ligand-1.

M2 macrophages facilitate wound healing, tissue repair, and remodeling after inflammatory injury (via factors such as TGF-β) and antagonize the action of macrophages (mediated by IL-10) [37,38]. This reflects the critical role of M2 macrophages as natural feedback regulators of the inflammatory process. The balance between M1 and M2 macrophages is critical for homeostasis. An increased M1/M2 macrophage ratio results in severe inflammation and tissue damage, and a decreased ratio leads to tissue and organ fibrosis [27].

High-throughput technologies such as single-cell sequencing technology are changing the classical definition of macrophage subpopulations [39,40]. There are a mushrooming number of classification markers for macrophage subpopulations, and there may be shared markers between subpopulations. The concept of mixed phenotypes begins budding. But currently, there are not many studies on mixed phenotypes in SSc, and future studies may focus more precisely on classified macrophage populations to reveal more distinct lineages of monocytes/macrophages and their role in fibrosis in SSc.

### 2.3 M2 macrophages in SSc

Macrophages are a heterogeneous class of cells that play a key role in inflammation and tissue repair, but abnormal activation of macrophages may lead to chronic inflammation and tissue fibrosis [41,42]. As described in the previous section, chronic inflammation is the main culprit of SSc tissue fibrosis, which has led researchers to associate macrophages with SSc fibrosis. An analysis of skin biopsy RNA sequencing data from 48 SSc patients and 33 matched healthy controls (HCs) showed that the most common upregulated signatures in SSc compared to HCs were M2 and M1 cells (96% and 94% of SSc patients, respectively) and that macrophage-type characteristic was associated with a higher modified Rodnan skin score (mRSS) [43]. CD163 is one of the marker genes of M2 macrophages, plasma and urine samples from SSc patients contained significantly higher levels of sCD163 than HCs [44]; Compared to M1 macrophages, M2 macrophages secrete a large number of pro-fibrotic molecules such as TGF-β and VEGF (Fig. 2), which makes us shift our focus to M2 macrophages. A recent study found elevated percentages of monocytes/macrophages in the mixed M1/M2 phenotype in peripheral blood of patients with SSc [45], which is related with SSc-related interstitial lung disease (SSc-ILD) [46]; However, Flow assay results from SSc patients and HCs circulating cell showed significantly elevated M1 and M2 macrophage surface markers compared to HCs, no difference when only M1 markers were detected [47]; Meanwhile, gene-gene interaction networks created based on three transcriptomic datasets from SSc skin biopsies showed that M2 macrophage activation is the core molecular process in the SSc molecular network [48]. Given the close association of M2 macrophages with SSc fibrosis, we summarize the inhibitors of M2 macrophage polarization that ameliorate SSc and the role of M2 macrophages in SSc.

## 3 Molecular mechanism and targeted therapy of M2 polarization in different organ fibrotic lesions

### 3.1 Skin fibrosis

The most prominent symptoms of SSc are skin fibrosis and hardness [49], The extent of skin involvement and its rate of progression is associated with internal organ involvement, dysfunction, and survival [50]. Multiple studies link SSc skin fibrosis with M2 macrophages. *N*-acetylglucosamine aminotransferase V (GNT-V) is highly expressed in M2 macrophages in SSc skin samples, and knockout of GNT-V in bleomycin (BLM)-induced SSc mouse model dramatically reduced CD163^+^M2 macrophages, dermal thickness, and collagen 1α1 expression [51]. Compared with wild-type (WT) mice, BLM induced more severe skin fibrosis in *Fli-1*^*+/−*^ mice, and macrophages in *Fli-1*^*+/−*^ mice were treated with interleukin-4 (IL-4) or IL-13 stimulation with preferential differentiation to M2 phenotype [52]. Levels of the transcriptional regulator IRF8 were significantly suppressed in monocytes from patients with diffuse cutaneous SSc and negatively correlated with the mRSS, and IRF8-silenced monocyte-derived macrophages displayed an M2 phenotype and significantly Along with upregulating the mRNA and protein levels of pro-fibrotic factors and extracellular matrix components, IRF8 silencing also exhibited a pro-fibrotic trend in a BLM-induced fibrosis mouse model [53]. According to recent studies, some inhibitors of M2 polarization manifest antifibrotic functions (Table 1).

**Table 1:** Inhibitors of M2 polarization and their anti-fibrotic mechanisms in mouse models of skin fibrosis.

Inhibitors	Mechanisms	References
CX3CL1mAb	Reduce the infiltration of M1 and M2 macrophages in the fibrotic skin as induced by TGF-β and CTGF.	[54]
DZ200	Suppress the expression of pro-inflammatory Th1, Th2, and Th17 cytokines and chemokines in BLM-induced fibrotic skin tissues, and inhibit the polarization of BMDMs to M1, and M2 macrophages. Regulate the TGF-β/Smad signaling pathway and relieve fibrosis.	[55]
Paquinimod	Induce the differentiation of M2 macrophages into M1 macrophages, reduce the reactivity of TGF-β and increase the production of autoantibodies in the fibrotic mouse model (Tsk-1), thereby reducing the number of myofibroblasts and the degree of fibrosis.	[56]
HPH-15	Resist the phosphorylation of Smad3 in human skin fibroblasts induced by TGF-β and inhibit the expression of α-SMA, COL1A2, FN1, and CTGF. improve the infiltration of M1 and M2 macrophages, in the BLM-induced fibrosis model, and prevent and effectively improve formed skin fibrosis.	[57]
WKYMVm	Improve the infiltration of M2 macrophages in the skin and reduce the levels of TNF-α and IFN-γ.	[58]
Glycyrrhizin	Inhibit the expression of Th2-related cytokines, thereby reducing the polarization and infiltration of M2 macrophages in BLM-induced fibrotic skin. Inhibit the activation of TGF-β-dependent dermal fibroblasts, thereby reducing the BLM-induced fibrosis effect.	[59]
Tocilizumab	Neutralize IL-6 and resist IL-6-induced M2 macrophage production.	[60,61]
Rolipram and apremilast	Rolipram and apremilast are phosphodiesterase 4 (PDE4) inhibitors. Inhibition of PDE4 suppresses the release of pro-fibrotic cytokines and the differentiation of M2 macrophages, thereby reducing the activation of fibroblasts and the release of collagen.	[62]

CX3CL1, Fractalkine/CX3C chemokine ligand 1; CTGF, connective tissue growth factor; DZ200, a reversible *S*-adenosyl-l-homocysteine hydrolase (SAHH) inhibitor; BMDMs, bone marrow-derived macrophages; HPH-15, histidine-pyridine-histidine ligand derivative; α-SMA, alpha-smooth muscle actin; COL1A2, collagen type I alpha 2; FN1, fibronectin 1.

### 3.2 Pulmonary fibrosis

M2 macrophages are significantly upregulated in BLM-induced mouse models of pulmonary fibrosis, SSc-ILD, and idiopathic pulmonary fibrosis (IPF), and are closely related to fibrosis progression [46,63,64]. However, currently, no clinically applicable therapy targets M2 macrophages to suppress pulmonary fibrosis. In BLM-induced pulmonary fibrosis, recent studies have shown that inhibitors of M2 polarization alleviated fibrosis (Table 2). In this section, we have summarized the regulatory mechanisms and potential inhibitors of M2 polarization in pulmonary fibrosis (Fig. 3).

**Table 2:** Inhibitors of M2 polarization in models of pulmonary fibrosis and their anti-fibrotic mechanisms.

Inhibitors	Mechanisms	References
JAK inhibitors	Down-regulate polarization markers (CD86, *MHC-II*, TLR4) and inflammatory cytokines (CXCL10, IL-6, TNF-α), and restrict the activation of M2 macrophages.	[65]
Nintedanib	Impair the polarization of monocytes towards M2 and reduce the number of M2 macrophages.	[66]
Pirfenidone	Reduce the expression of M2 markers and the release of TGF-β1 from M2 alveolar macrophages and attenuate the proliferation of lung fibroblasts from the culture supernatant of M2 alveolar macrophages.	[67]
Schisandra	Suppress the polarization of AM to M2 macrophages by inhibiting the TGF-β1/Smad pathway.	[68]
Microcystin-LR	Inhibit the endoplasmic reticulum stress response (Accumulation of misfolded proteins in the endoplasmic reticulum. This condition is called endoplasmic reticulum stress. The endoplasmic reticulum stress of macrophages in the lung may be beneficial to the polarization of M2 macrophages [69,70]) mediated by glucose regulatory protein 78 (GRP78).	[71]
Imatinib-loaded gold nanoparticles	Induce apoptosis in lung fibroblasts, inhibit their proliferation and viability and effectively limit IL-8 production, AM viability, and M2 polarization.	[72]

JAK, Janus kinase; *MHC-II*, *MHC* class *II*; TLR4, Toll-like receptor 4; CXCL10, C-X-C motif ligand 10.

**Fig. 3:** Mechanisms of M2 polarization in pulmonary fibrosis. Signal transducer and activator of transcription 3 (STAT3) and STAT6 are the most important participants in M2 polarization. Cytokines or other molecules drive M2 polarization by activating STAT3 and STAT6. MDB2, CpG binding domain 2; Start1, spliceosome associated factor 1; Cu, Zn-SOD, Cu, Zn-superoxide dismutase; Chop, C/EBP homologous protein; PPAR-γ, peroxisome proliferator-activated receptor-γ.

CpG-binding domain 2 (MBD2) and matrix metalloproteinase 28 (MMP28) are two proteins that promote M2 polarization in pulmonary fibrosis. MBD2 was significantly upregulated in both SSc-ILD and IPF, while MBD2 depletion attenuated BLM-induced lung fibrosis in mice and suppressed TGF-β production and M2 macrophage accumulation. Mechanistically, MDB2 selectively binds to the *Ship* promoter in macrophages, thereby suppressing Ship expression and heightening PI3K/Akt signaling to promote the macrophage M2 program [73]. MMP28 belongs to the matrix metalloproteinase family, and *Mmp28*^−/−^ M2 macrophages had a lower degree of polarization than WT cells during the M2 polarization triggered by IL-4 and IL-13. Simultaneously, *Mmp28*^−/−^ mice exhibited a reduced degree of fibrosis when BLM was induced [74].

Signal transducer and activator of transcription 3 (STAT3) and STAT6 are essential for the M2 program in macrophages. IL-4/IL-10 stimulation shifts alveolar macrophages to M2 macrophages in patients with fibrotic ILD by inducing activation of STAT3 [75]; IL-6 acts on IL-6 receptor alpha (IL-6Rα) bound to the surface membrane of macrophages, which activates STAT3 and promotes M2 polarization mediated by IL-4 and IL-13. Transient adenoviral IL-6 overexpression promotes M2-like macrophage accumulation and the development of fibrotic lung disease [76]. C/EBP homologous protein (CHOP) [77], spliceosome associated factor 1 (Sart1) [78], Cu, Zn-superoxide dismutase (Cu, Zn-SOD) [79], and long non-coding RNA (lncRNA)-MM2P [80] promote M2 polarization and BLM-induced fibrosis via STAT6 activation. CHOP is an endoplasmic reticulum (ER) stress marker. Loss of CHOP protected mice from lung injury and fibrosis induced by BLM and increased the expression of suppressors of cytokine signaling 1 (SOCS1) and SOCS3. SOCS1 and SOCS3 restrict M2 macrophage polarization and attenuate TGF-β1 expression in alveolar lavage fluid by repressing STAT6/PPAR-γ signaling. *CHOP*^*−/-*^ and BLM-induced WT mice developed equal degrees of fibrosis after clearing macrophages with neutral chlorophosphate liposomes, suggesting that CHOP causes pulmonary fibrosis by promoting M2 polarization [77]. Sart1 also promotes M2 polarization by activating STAT6/PPAR-γ, and siRNA-loaded liposomes targeting Sart1 significantly attenuate M2 macrophage polarization by blocking the STAT6/PPAR-γ signaling axis. Simultaneously, intratracheal administration of siRNA-loaded liposomes targeting Sart1 significantly suppressed BLM-induced pulmonary fibrosis [78]. By redox-regulating, a crucial cysteine in STAT6, Cu, Zn-SOD modulates H2O2 levels that modulate M2 gene expression at the transcriptional level, polarizing macrophages to an M2 phenotype. Additionally, Cu, Zn-SOD overexpression in mice causes a pro-fibrotic environment and accelerates the progression of pulmonary fibrosis [79]. Long non-coding RNAs (lncRNAs) are involved in the regulation of immune cell differentiation and function. The only lncRNA that was upregulated during M2 polarization and downregulated in M1 macrophages, according to the results of the lncRNA chip analysis of the M2 macrophage polarization model, was lncRNA-MM2P. Furthermore, inhibiting lncRNA-MM2P blocks cytokine-driven M2 polarization and represses the proangiogenic function of M2 macrophages by decreasing STAT6 phosphorylation [80].

It is believed that STAT6 acetylation is a crucially important negative regulatory mechanism that prevents macrophage M2 polarization. By accelerating the CREB-binding protein (CBP)'s ubiquitination at Lys119, Trim24, an E3 ligase connected to CBP, makes it easier for CBP to bind to STAT6. Trim24 loss reduces STAT6 acetylation in both mouse and human macrophages, which in turn promotes M2 polarization [81]. This study was not performed in a pulmonary fibrosis model, nevertheless, it is a novel addition to the M2 macrophage polarization mechanism.

Taken together, these studies offer a possible therapeutic target for hindering the accelerated progression of pulmonary fibrosis and offer novel treatments, such as the intratracheal administration of siRNA-loaded liposomes. In the future, siRNA-loaded liposomes may become the mainstream therapy for targeting pathogenic factors.

### 3.3 Cardiac fibrosis

The most common cause of death in SSc patients is now cardiomyopathy, surpassing cancer in this regard. An autopsy of myocardial histology in patients with SSc with no clinical symptoms of cardiac involvement revealed that all patients had cardiomyopathy [82]. Abnormal fibrosis of the myocardial tissue is a prominent aspect of SSc cardiac performance; however, symptoms may not be detected for a long period. Cardiac insufficiency, such as lower ventricular ejection fraction caused by systolic and diastolic dysfunction, occurs late in SSc. Myocardial fibrosis in SSc affects the ventricular walls and impairs the relaxation of myocardial tissue during diastole [83]. Previous studies have shown that M2 macrophages are actively involved in myocardial fibrosis caused by other diseases. Excessive M2 macrophage infiltration in the atrial tissue of patients with atrial fibrillation is positively correlated with myocardial fibrosis and collagen gene expression [84]. M2 macrophages are involved in the progression of hypertrophic cardiomyopathy (HCM). Inhibition of M2 macrophage polarization effectively reduces the degree of cardiac fibrosis [85]. These findings suggest that M2 macrophages play a role in cardiac fibrosis. Future studies may find evidence that M2 macrophages are involved in cardiac fibrosis in SSc.

## 4 Mechanisms of M2 macrophage regulation of fibrosis

One of the key causes of excessive matrix accumulation is the survival of metabolically active, apoptosis-resistant myofibroblasts.α-SMA-expressing myofibroblasts are derived from a variety of stromal progenitor cell types, such as fibroblasts, pericytes, and ECs [17]. Fibroblast subtypes defined based on differential expression of gene modules and signaling pathways, pointing to diverse functions including skin maintenance, ECM remodeling, fibrosis, and immune regulation [9], fibroblast crosstalk with other cells, may lead to its transition to a profibrotic subtype. Research has shown that M2 macrophages promote fibrosis by driving epithelial-mesenchymal transition (EMT) and fibroblast-myofibroblast transition (FMT) through the secretion of fibrogenic mediators, particularly TGF-β1. The TGF-β/Smad and Wnt/β-catenin signaling pathways are essential in the progression of M2 macrophage-induced fibrosis (Fig. 4).

**Fig. 4:** Mechanisms of M2 macrophage regulation of fibrosis. M2 macrophages produce and secrete pro-fibrotic cytokines or proteins, which activate TGF-β/Smad signaling or Wnt/β-catenin to facilitate the epithelial-mesenchymal transition and fibroblast-myofibroblast transition. Non-coding RNAs, including lncRNAs and miRNAs, also contribute to fibrosis in which M2 macrophages are involved.

### 4.1 Driving EMT

EMT is a phenotypic transformation of differentiated epithelial cells into myofibroblasts capable of producing ECM, and it is widely regarded as an essential component of fibrogenesis following tissue injury [86]. EMT and its intermediate states have recently been identified as crucial drivers of argan fibrosis and tumor progression. Recent research has suggested that M2 macrophages are closely linked to EMT [71,87].

TGF-β is a multifunctional cytokine that is essential for fibrosis induction. Overexpression of TGF-β causes EMT, ECM deposition, and cancer-associated fibroblast formation, leading to fibrotic diseases and cancer. The development of fibrosis depends heavily on TGF-β and its associated molecules [88]. *In vitro* experiments demonstrated that M2 macrophages produce a large quantity of TGF-β, upregulate α-SMA expression, and decrease E-cadherin expression in lung epithelial cells. In this process, the TGF-β/Smad2 signaling pathway is activated, and it is repressed after treatment with TGF receptor inhibitors and EMT is blocked [87,89]. Other molecules activated by TGF-β are also involved in the EMT. LncRNAs are important signal transduction regulators that act on various patterns. By competitively binding to the miR-200 family, lncRNA-ATB triggers EMT in various malignancies. TGF-β induces lncRNA-ATB expression in pulmonary epithelial cells and induces EMT. lncRNA-ATB acts as a miR-200c sponge to diminish the repressive effect of miR-200c on ZEB1, which is a mesenchymal marker [90]. ZEB1 regulates E-cadherin expression and EMT by repressing many master regulators of epithelial polarity [91]. Thus, the mechanism by which M2 macrophages promote EMT is, at least in part, due to the activation of TGF-β/Smad signaling.

### 4.2 Driving FMT

Fibroblast activation is the final step in the pathophysiology of SSc. A substantial number of α-SMA-positive myofibroblasts produce excessive ECM in the involved organs, resulting in fibrosis and sclerosis [92]. Myofibroblasts are key effector cells in ECM remodeling in SSc-related fibrosis, and FMT is widely recognized as the major pathological feature of multiple organ fibrosis. By driving FMT, M2 macrophages promote the progression of fibrosis in the lesion organs.

TGF-β and PDGF, which are generated and secreted by M2 macrophages, are critical pro-fibrotic cytokines involved in fibroblast activation. TGF-β stimulates the expression of DNA methyltransferase 1 (DNMT1) and DNMT3A in fibroblasts in a Smad-dependent manner in fibrotic skin of patients with SSc and suppresses SOCS3 through promoter methylation. Downregulation of SOCS3 activates STAT3, thereby promoting the conversion of fibroblasts to myofibroblasts, collagen release, and fibrosis *in vitro* and *in vivo* [93]. Besides TGF-β, platelet-derived growth factor-CC (PDGF-CC) secreted by M2 macrophages can upregulate α-SMA in the dermis, which is a classical symbol of myofibroblasts [94]. M2 macrophages also express high levels of Wnt7a, which induces the activation of the Wnt/β-catenin signaling pathway, leading to lung resident mesenchymal stem cells (LR-MSC) differentiating into myofibroblasts; conversely, blocking the Wnt/β-catenin signaling pathway inhibits BLM-induced pulmonary fibrosis [63]. miRNAs are post-transcriptional repressors of gene function and are small non-coding RNAs of approximately 22 nucleotides [95]. Exosomal miR-328 downregulates FAM13A, a susceptibility gene for chronic obstructive pulmonary disease. Exosomes derived from M2 macrophage that overexpress miR-328 exacerbate pulmonary fibrosis by silencing FAM13A [96]. The proteins secreted by M2 macrophages may also play a role in fibroblast regulation. S100a4, also known as fibroblast-specific protein 1 (FSP-1), was once thought to be a fibroblast marker that promotes lung fibroblast proliferation and activation [97].

## 5 Conclusion

In summary, M2 polarization is the culprit and is at least partly responsible for the progression of SSc fibrosis. Pro-fibrotic cytokines produced and secreted by M2 macrophages drive both EMT and FMT, both of which contribute to the progression of fibrosis. Understanding the mechanisms of M2 polarization in SSc and how M2 macrophages are involved in fibrosis could provide new options for fibrosis treatment. Studies carried out on fibrosis in animal models have found that *anti*-M2 polarization and infiltration could effectively alleviate fibrosis, suggesting that *anti*-M2 macrophage strategies could offer promising strategies for treating SSc fibrosis and other fibrosis-related disorders.

## Author contribution statement

All authors listed have significantly contributed to the development and the writing of this article.

## Data availability statement

No data was used for the research described in the article.

## Declaration of competing interest

The authors declare that they have no known competing financial interests or personal relationships that could have appeared to influence the work reported in this paper.
